RETRACTED

# The Mechanism of Xiaoyao San in the Treatment of Ovarian Cancer by Network Pharmacology and the Effect of Stigmasterol on the PI3K/Akt Pathway

**DOI:** 10.1155/2021/4304507

**Published:** 2021-06-29

**Authors:** Meng Li, Wenqi Zhang, Linqi Yang, Huibing Wang, Yihan Wang, Kai Huang, Wei Zhang

**Affiliations:** ^1^Department of Pharmacology, College of Basic Medicine, Hebei University of Chinese Medicine, Shijiazhuang, 050200 Hebei Province, China; ^2^Department of Hematology, The Fourth Hospital of Hebei Medical University, Shijiazhuang, 050000 Hebei Province, China

## Abstract

**Purpose:**

This study was aimed at exploring the regulatory mechanism of Xiaoyao San (XYS) and its main compound, Stigmasterol, in the biological network and signaling pathway of ovarian cancer (OC) through network pharmacology-based analyses and experimental validation.

**Methods:**

The active compounds and targets of XYS were studied by the Traditional Chinese Medicine Systems Pharmacology Database and Analysis Platform (TCMSP). The GeneCards and OMIM databases were used to screen common targets of XYS in the treatment of OC. Combined with the STRING database and Cytoscape 3.6.0, the core compounds and targets of XYS were obtained. GO and KEGG pathway enrichment analyses of core target genes were carried out by using the Metascape and DAVID databases. Molecular docking has been achieved by using the AutoDock Vina program to discuss the interaction of the core targets and compounds of XYS in the treatment of OC. The effect of Stigmasterol on proliferation and migration were assessed by CCK8 and wound healing assay. Western blot and qRT-PCR were used to analyze the protein and mRNA expressions of PI3K, Akt, and PTEN after treatment of Stigmasterol.

**Results:**

A total of 113 common targets of XYS for the treatment of OC were obtained from 975 targets related to OC and 239 targets of XYS's effect. The main compounds of XYS include Quercetin, Naringenin, Isorhamnetin, and Stigmasterol, which mainly regulate the targets such as TP53, Akt1, and MYC and PI3K/Akt, p53, and cell cycle signal pathways. At the same time, molecular docking showed that Stigmasterol and Akt1 had good docking conformation. Stigmasterol inhibited OC cell proliferation and migration in vitro and reduced the protein and mRNA expressions of the PI3K/Akt signaling pathway.

**Conclusion:**

Stigmasterol as the one of the main compounds of XYS suppresses OC cell activities through the PI3K-Akt signaling pathway.

## 1. Introduction

Ovarian cancer (OC) is the most frequently diagnosed and highest mortality in gynecological cancers. The 5-year overall survival rate was about 40% when most patients were late at the time of discovery because the lack of symptoms was not obvious [1, 2]. Currently, the main treatment of OC is surgery, platinum-based chemotherapy, and radiotherapy. In a clinical study, 30-45% BRCA1/2 mutation patients showed response to the PARP inhibitor Olaparib. But relapse and metastasis were considered to be due to resistance and toxicities. Therefore, how to increase the response rate and relieve side effects still remains to be completed. A number of clinical trials have shown that the traditional Chinese medicine combination with chemotherapy or radiotherapy may benefit OC patients [3–5].

RETRACTED

XYS from Prescriptions of Peaceful Benevolent Dispensary can soothe the liver, nourish the blood, invigorate the spleen, and harmonize the heart. It is mostly used for hepatic stagnation, spleen deficiency, and blood deficiency syndrome. However, the mechanism of XYS in the treatment of OC is unknown and needs further discussion.

With the rapid development of bioinformatics, systems biology, and polypharmacology, network-based drug discovery is considered to be an economical and effective drug development method [6]. In recent years, increasing evidence has shown that many drugs can stimulate their therapeutic activities by regulating multiple targets [7]. Due to the abundant ingredients in Chinese herbs and the complex changes of disease-related molecules, the mechanism of most traditional Chinese medicines (TCM) and their derivatives in complex diseases remains to be elucidated.

In this study, several drug target prediction databases were used to analyze XYS, and the protein-protein interaction network (PPI) of the main targets of XYS in the treatment of OC was constructed to explore its main biological functions and signaling pathways. Finally, the effect of Stigmasterol on the PI3K/Akt signaling pathway was verified by a cell experiment in vitro, which provides a new basis for the development and application of XYS and its compound Stigmasterol.

## 2. Materials and Methods

### 2.1. Main Drugs and Reagents

Fetal bovine serum (FBS) was obtained from HyClone (USA), and RPMI (Roswell Park Memorial Institute) 1640 medium, penicillin, streptomycin, and all other reagents were obtained from GIBCO (USA). Stigmasterol (purity: 98%, APExBIO Technology LLC) was dissolved in DMSO and stored at -20°C. The final concentration of DMSO in cultures was ≤0.1% (*v*/*v*).

### 2.2. Common Targets of XYS in the Treatment of OC

The Traditional Chinese Medicine Systems Pharmacology Database and Analysis Platform (TCMSP, http://www.tcmspw.com/tcmsp.php) was used to collect the active compounds of XYS, including Bupleurum, Radix Paeoniae Alba, Angelica sinensis, Atractylodes macrocephala, Poria cocos, Glycyrrhiza uralensis, ginger, and peppermint. The active compounds and their targets in the composition of XYS were selected by ADME evaluation systems, the main parameters of which were oral bioavailability (OB ≥ 30%) and drug-likeness (DL ≥ 0.18). Through the STRING database (https://string-db.org/) [8], the collected target names of XYS were standardized gene IDs, and species sources were humans (“Homo sapiens”). GeneCards (https://www.genecards.org/) and OMIM (https://omim.org/) were utilized to collect genes and targets related with OC [9]. The 113 common targets of OC and active components were obtained by Draw Venn Diagram (http://bioinformatics.psb.ugent.be/webtools/Venn/) (Figure 1).

RETRACTED

### 2.3. Protein-Protein Interaction (PPI) Network

The PPI network was obtained from the above 113 common targets by STRING and “Homo species” was selected. The minimum interaction threshold was selected as “medium confidence >0.4.” The Cytoscape 3.6.0 software was used to analyze the core targets of the network, and “PNG” format was the output (Figure 1). The top 3 targets (TP53, Akt1, MYC) were identified as the hub genes of XYS in the treatment of OC, which were used in following studies. The expressions of the top 3 targets were acquired in https://www.helixlife.cn/.

### 2.4. Gene Ontology (GO) and Kyoto Encyclopedia of Genes and Genomes (KEGG) Pathway Enrichment Analyses

The GO and KEGG enrichment analyses were obtained from the above 113 common targets by the Metascape database (http://metascape.org/) and DAVID database (https://david.ncifcrf.gov/); *P* < 0.05 was significant.

### 2.5. Construction of Herb-Active Compound-Target Network

Cytoscape 3.6.0 was used to construct the “herb-active compound-target” network of XYS in the treatment of OC. We identify the top 10 active compounds as the core compounds of XYS in the treatment of OC.

### 2.6. Molecular Docking

The interaction between the core compounds and targets of XYS in the treatment of OC was checked by using molecular docking technology. The target protein structures were downloaded from the PDB website (http://www.rcsb.org/), and the 3D structures of the core compounds were downloaded from the TCMSP database. The molecular docking and conformation scoring were carried out in the AutoDock Vina.

The heat map was obtained by the GraphPad Prism 8. The PyMOL and Maestro 11.9 were used to draw the structure of the best docking results.

### 2.7. Relationship between the mRNA Levels of Akt1 and the Survival Outcomes of Patients with OC

We utilized R3.6.3 software to carry out the receiver operating characteristic curve (ROC curve) and Kaplan-Meier curve (KM curve) enrichment analyses. We prepared the RNAseq data and clinical data from the ovarian serous cystadenocarcinoma (OV) project in TCGA (https://portal.gdc.cancer.gov/) and transformed them into transcripts per million read (TPM) format and then analyzed them according to the molecular expression.

RETRACTED

### 2.8. Culture of OC Cell Lines

A2780 and SKOV3 cell lines were cultured in RPMI1640 medium with 10% (*v*/*v*) FBS and 100 U/ml penicillin/100 mg/ml streptomycin at 37°C in the 5% CO_2_ atmosphere.

### 2.9. Cell Proliferation Assay

Ovarian cancer A2780 and SKOV3 cells were seeded into 96-well plates with gradient concentration (0 *μ*M, 10 *μ*M, 25 *μ*M, 50 *μ*M, 100 *μ*M, and 500 *μ*M) Stigmasterol for 24, 48, and 72 hours at 37°C. The OC cells were replaced with a 10% Cell Counting Kit-8 (CCK8; Beijing Zoman Biotechnology Co., Ltd., Beijing, China) diluted with normal culture medium and incubated for 1 h. The absorbance of each well was measured with a Motic digital medical image analysis system (Leica DM2500, Heidelberg, Germany) at 450 nm. All tests were repeated three times [10].

### 2.10. Preparation of Stigmasterol

Stigmasterol was dissolved in DMSO, mixed and filtered through a 0.22 *μ*m filter. The stock solution at 10 mM concentration was prepared and stored in a refrigerator at -20°C, and it was defrosted and diluted to the desired concentration with 1640 complete medium before use.

### 2.11. Wound Healing Assay

The comparison of the cell culture area for the wound-healing assay was generated by a 10 *μ*l pipette tip, after A2780 and SKOV3 cells were cultured in the RPMI1640 medium with 10% FBS without or with 25 and 50 *μ*M Stigmasterol, respectively. The Motic digital medical image analysis system was used by Leica DM2500, Heidelberg, Germany [11].

### 2.12. Real-Time Fluorescence Quantitative Polymerase Chain Reaction (qRT-PCR)

Total RNA from the above-mentioned cells was isolated with a TRIzol Reagent (Life Technologies, USA) according to the manufacturer's instructions. RNA concentration and purity were assessed by spectrophotometry at 260 nm. A total of 1 *μ*g RNA was converted into cDNA by a Prime Script RT reagent Kit (Takara Co. Ltd., USA). qRT-PCR was performed by using a Real-Time PCR System (Bio-Rad Co. Ltd., USA) in reaction mixtures (25 *μ*l) containing cDNA, primer pairs (Table 1), and TB Green Premix Ex Taq II (Takara Co. Ltd., USA).

### 2.13. Western Blot (WB)

A2780 and SKOV3 cells were treated with Stigmasterol for 48 h. After washing with PBS three times, the cells were lysed for 30 min on ice and centrifuged at 10000 × g for 5 min at 4°C. The contents of segregated proteins in cell lysates were quantified using an ND-1000 Spectrophotometer (NanoDrop, Wilmington, Delaware, USA). Equal amounts of protein samples were electrophoresed through 10% SDS-PAGE (polyacrylamide gel electrophoresis) and transferred to PVDF membranes (Millipore, Bedford, Massachusetts, USA). After 5% BSA block for 2 h, they were immunoblotted with primary antibodies for overnight at 4°C. The primary antibodies include p-Akt (GB13012-3, 1 : 500), Akt (GTX28805, 1 : 800), p-PI3K (GTX132597, 1 : 800), PI3K (ab40755, 1 : 1000), PTEN (ET1606-43, 1 : 800), and *β*-actin (AC026, 1 : 10000). Next, the membranes were incubated with secondary antibodies of goat anti-rabbit IG (KPL074-1506, at 1 : 5000 dilution) for 1 h at 37°C. The intensity of protein bands was estimated via executing the Fusion FX5 Spectra (Fusion, France).

RETRACTED

## 3. Results

### 3.1. PPI Network of XYS in Treatment of OC

In Figure 1, the XYS in the treatment of the OC interaction network with 113 nodes and 1805 edges is shown. The Cytoscape was adopted to obtain the top 3 hub targets of interactions including TP53, Akt1, and MYC. As a result, the expression of Akt1 and TP53 was higher and that of MYC was lower in OC tissues than in normal tissues (Figure 1).

### 3.2. GO and KEGG Pathway Enrichment Analyses

The GO and KEGG pathway of targets of XYS in the treatment of OC were involved in 338 signaling pathways, including the PI3K-Akt signaling pathway, bladder cancer, pancreatic cancer, hepatitis B, microRNAs in cancer, and HIF-1 signaling pathway. The top 20 pathways are shown in Figure 2.

### 3.3. Herb-Active Compound-Target Network

This network graph directly evaluates the mechanism of XYS in the treatment of OC through multicompound and multitarget synergistic action. The herb-active compound-target network has shown the top 10 active compounds of XYS in the treatment of OC including Quercetin, Kaempferol, and Stigmasterol (Table 2).

### 3.4. Molecular Docking

The top 10 main compounds of XYS were docked with the protein structures of Akt1, TP53, and MYC. The results showed that Stigmasterol was the best binding ability to Akt1 and the Vina score (ΔG) was -10.60 kca1/mol (Figure 2). The molecular docking revealed the Stigmasterol bond with Akt1 through hydrophobic interaction at sites such as LEU264, VAL270, LEU210, and LEU264 (Figure 2).

### 3.5. Relationship between the mRNA Levels of Akt1 and the Survival Outcomes of Patients with OC

We further explored the critical efficiency of Akt1 in the survival of patients with OC. The ROC curve analysis for Akt1 in OC determined that AUC of the ROC curve is 0.702. The Kaplan–Meier curve and log-rank test analysis revealed that the increased Akt1 mRNA levels were significantly associated with the overall survival (OS) of OC patients (Figure 2). Higher expression of Akt1 showed the longer overall survival.

RETRACTED

### 3.6. Effect of Stigmasterol on the Proliferation of A2780 and SKOV3 Cells

The CCK8 assay result suggested that Stigmasterol could significantly inhibit A2780 and SKOV3 cell proliferation in a dose-dependent manner (*P* < 0.05). The IC_50_ values are shown in Table 3. The following experiments were carried out with Stigmasterol at concentrations of 25 *μ*M and 50 *μ*M for 48 h.

### 3.7. Effect of Stigmasterol on the Migration of A2780 and SKOV3 Cells

As the result of compound Stigmasterol displayed a significant cytotoxic activity against ovarian cancer A2780 and SKOV3 cell lines, the wound healing assay showed that Stigmasterol inhibited migration of A2780 and SKOV3 cells (Figure 3).

### 3.8. Stigmasterol Inhibited the mRNA Expression of PI3K-Akt Signaling Pathway in A2780 and SKOV3 Cell Lines by qRT-PCR

The results of qRT-PCR showed that comparing with the control and DMSO groups, the mRNA expression of PI3K and Akt1 was significantly reduced by Stigmasterol. The mRNA expression of PTEN was increased in Stigmasterol groups (*P* < 0.05) (Figure 3).

### 3.9. Stigmasterol Inhibited the Protein Expression of PI3K-Akt Signaling Pathway in A2780 and SKOV3 Cell Lines by Western Blot Assay

The protein expressions of p-PI3K/PI3K and p-Akt/Akt were significantly decreased, and the PTEN expression was increased in Stigmasterol groups compared with the control and DMSO groups (*P* < 0.05) (Figure 3). This result showed that Stigmasterol can effectively inhibit the PI3K-Akt signaling pathway in human A2780 and SKOV3 cells.

## 4. Discussion

In traditional Chinese medicine, XYS has been proposed for anticancer activities and was used in the treatment of breast hyperplasia, breast cancer, and OC by reinforcing qi and nourishing the blood. XYS is a classic Chinese prescription which was first described in the Prescriptions of Peaceful Benevolent Dispensary in the Song Dynasty (A.D. 1151).

In this study, as the result of the network pharmacology, XYS possessed the multicomponent, multitarget synergistic effect in the treatment of OC. The main active compounds of XYS in this network include Quercetin, *β*-sitosterol, Kaempferol, and Stigmasterol. Previous studies indicated that Quercetin has the anticancer activities involved in downregulating the levels of RAS, BCL-2, mutant P53, and upregulating BAX [12]. Studies have shown that *β*-sitosterol has the wide anticancer properties such as inducing apoptosis and inhibiting proliferation, invasion, metastasis, and angiogenesis in colon cancer, ovarian cancer, lung cancer, breast cancer, and prostate cancer. *β*-Sitosterol exerted against ovarian cancers by estrogen reabsorption. Also, *β*-sitosterol decreased the expression of *β*-catenin, PCNA (proliferating cell nuclear antigen), and Bcl-2 in colon cancer [13]. Kaempferol can reduce the expressions of p-Akt (phosphorylated Akt) protein in OC cells. It inhibits cell migration and angiogenesis in human OC cells, induces apoptosis and ROS production, and thus inhibits the growth and development of human OC cells [14]; Stigmasterol effectively targets tumor endothelial cells by suppressing the expressions of TNF-2, VEGFR-2 and p-Akt, PCL, and FAK [15].

RETRACTED

The PPI network of XYS in the treatment of OC indicated that the core targets include Akt1, TP53, and MYC. Therefore, we used the database to analyze the expression of the above 3 hub genes in OC tissues and normal tissues. The results showed that Akt1 and TP53 were highly expressed in OC tissues and MYC expression was lower in OC tissues than in normal tissues. GO and KEGG pathway enrichment analyses of XYS in the treatment of OC also found that the PI3K/Akt signaling pathway plays a role in OC signaling pathways. From the molecular docking result, Stigmasterol showed a strong interaction with Akt1. Meanwhile, the expression of Akt1 in OC is closely related to OS of clinical patients. Therefore, we predict that Akt1 may be a potential core target of Stigmasterol for the treatment of OC.

In clinical researches, the dysregulations of the PI3K/Akt signaling pathway were found in 70% OC, involving PTEN deletion and PIK3CA mutations [16]. Genetic alterations and aberrant activation of AKT are due to the ovarian cell carcinoma. Some researches showed that the AKT pathway was involved in cancer cell migration, invasion, and autophagy, which was considered as the potential therapeutic targets in the treatment of OC [16–19]. PI3K/Akt/mTOR pathway inhibitors become new tumor target drugs in OC clinical applicability [18].

Based on these results, we further verified the effect of Stigmasterol on the PI3K-Akt signaling pathway in OC cell lines A2780 and SKOV3. According to the results of the CCK8 assay and the wound healing assay, the effect of Stigmasterol could significantly inhibit the proliferation and migration in A2780 and SKOV3 cells. Furthermore, Stigmasterol can reduce the levels of PI3K and Akt and increase the expression of PTEN in A2780 and SKOV3 cells. This research not only provides a theoretical and experimental basis for more in-depth studies but also offers an efficient method for the rational utilization of a series of Chinese medicine's active ingredients as anti-tumor drugs.

## 5. Conclusion

In summary, Stigmasterol, as the main active compound of XYS, could predict a candidate compound in OC therapy by targeting the PI3K/Akt signaling pathway.

RETRACTED

## Figures and Tables

**Figure 1:** (a) The targets of XYS in treatment of OC. Venn diagram showing 975 targets associated with OC and 239 targets of XYS. Overlap represents 113 common target genes. (b) The high expression of Akt1 and TP53 and low expression of MYC in OC. ^∗∗^*P* < 0.01, ^∗∗∗^*P* < 0.001. (c) Interaction target network of XYS treatment of OC. The top 3 targets in terms of degree value are TP53, Akt1, and MYC.

**Figure 2:** (a) GO enrichment in targets of XYS treatment of OC. (b) Top 20 of KEGG pathway enrichment in targets of XYS treatment of OC. (c) Results of molecular docking. Diagram of interaction between Akt1 protein and Stigmasterol (3D). (d) Relationship between the mRNA levels of Akt1 and the survival outcomes of patients with OC. A is the ROC curve of Akt1 in OC. B is the KM curve of Akt1 in OC.

**Figure 3:** (a) Stigmasterol inhibited the migration in A2780 cells. (b) The effect of Stigmasterol on expressions of the PI3K-Akt signaling pathway by qRT-PCR in A2780 cells. (c, d) Western blot assay showed that Stigmasterol downregulated the expression of p-PI3K and p-Akt protein levels and upregulated the expression of PI3K, Akt, and PTEN protein levels in A2780 cells. (e) Stigmasterol inhibited the migration in SKOV3 cells. (f) The effect of Stigmasterol on expressions of the PI3K-Akt signaling pathway by qRT-PCR in SKOV3 cells. The effect of Stigmasterol on expression of the PI3K-Akt signaling pathway in SKOV3 cells. Stigmasterol increased the mRNA expression level of PTEN and decreased the mRNA expression level of PI3K and Akt. (g, h) Western blot assay showed that Stigmasterol downregulated the expression of p-PI3K and p-Akt protein levels and upregulated the expression of PI3K, Akt, and PTEN protein levels in SKOV3 cells. ^∗^*P* < 0.05, ^∗∗^*P* < 0.01 vs. control group. The dosage of Stigmasterol was 25 *μ*M and 50 *μ*M in A2780 and SKOV3 cells, respectively.

**Table 1:** The primers of genes.

Primers	Forward (5′-3′)	Reverse (5′-3′)
PI3K	AGTAGGCAACCGTGAAGAAAAG	GAGGTGAATTGAGGTCCCTAAGA
AKT	AGCGACGTGGCTATTGTGAAG	GCCATCATTCTTGAGGAGGAAGT
PTEN	TGGATTCGACTTAGACTTGACCT	GGTGGGTTATGGTCTTCAAAAGG
*β*-Actin	TGACGTGGACATCCGCAAAG	CTGGAAGGTGGACAGCGAGG

**Table 2:** The top 10 active compounds of XYS in the treatment of OC.

No.	Active compounds
1	Quercetin
2	Kaempferol
3	Stigmasterol
4	Beta-sitosterol
5	Naringenin
6	Isorhamnetin
7	Luteolin
8	Formononetin
9	Licochalcone A
10	Medicarpin

**Table 3:** IC_50_ of Stigmasterol on A2780 and SKOV3 cells.

Time (hour)	IC_50_ (*μ*M) (mean ± SD)	
	A2780	SKOV3
24	69.24 ± 7.31	83.39 ± 3.75
48	49.74 ± 3.18	77.68 ± 5.43
72	38.12 ± 4.69	67.02 ± 3.13

RETRACTED

## Data Availability

The data are available upon direct request to the corresponding author.
